RETRACTED

# Data Fusion Algorithm for Myocardial Proteomics and Its Research in Sports

**DOI:** 10.1155/2022/4049169

**Published:** 2022-02-10

**Authors:** Ditao Song, Xiaoyong Hu

**Affiliations:** ^1^College of Physical Education, Guangxi Science & Technology Normal University, Laibin, 546199 Guangxi, China; ^2^Institute of Physical Education, Guiyang College, Guiyang, 550005 Guizhou, China

## Abstract

Sport is a type of comprehensive activity that the human body consciously engages in to improve physical fitness. Proteomics is a comprehensive technology dedicated to the study of all protein profiles expressed by a species, individual organ, tissue, or cell under specific conditions and specific times. Proteomics is a science that studies the protein composition of cells, tissues, or organisms and their changing laws with proteomics as the research object. Related technologies are now widely used in sports and other fields. The purpose of this article is to study myocardial proteomic technology and its application in sports. During the research process, the main methods used in this study are literature survey and controlled experiment. The results achieved and the problems in this field, followed by selecting 30 SD rats into 3 groups for control experiments. The results of the study showed that among the three groups of rats, the left ventricular ejection fraction of the sham operation group was the highest, which was 7.7% and 4.6% higher than that of the operation group and the model group, respectively. The operation group had the highest left ventricular short axis shortening rate, and the left ventricle diastolic inner diameter is the longest. It can be seen that myocardial proteomics can accurately reflect the heart condition of rats. In addition, the length, diastolic velocity, and diastolic time of cardiomyocytes of the three groups of rats were different. Among them, the cardiomyocytes of the operation group had the longest time and the longest diastolic time, which were 37.1% and 8.5% higher than those of the sham operation group and the model group.

## 1. Introduction

Sports are a comprehensive activity carried out by the human body consciously for improving physical fitness. Sports will bring a series of stimulations to the human body, such as muscle and nerve stimulation. The study of molecular mechanisms related to sports stimulation is a new trend in the field of exercise physiology that has caused the human body to respond and adapt in recent years. Sports will also cause a series of changes in the internal environment of the human body, which in turn affects the expression of related genes in other tissues and the synthesis of related proteins before and after exercise. Proteomics studies the characteristic expression of proteins in various biological samples at a large scale, which can serve to search for disease-specific proteins and take the corresponding intervention and treatment methods before patients appear onset symptoms. In the era of big data, proteomic data has undoubtedly become an important part of understanding the “whole” of life. Proteomic techniques and methods can be applied to explore the differences in the proteome of different organs and tissues in the human body under physical exercise conditions and therefore have become an important way to study the human body's response to exercise and the molecular biological mechanisms of exercise.

RETRACTED

In the clinical diagnosis and treatment of major human diseases such as cancer, Alzheimer's disease, and diabetes, proteomic technology has very broad application prospects. It can also provide an important basis for the early diagnosis of related diseases, the discovery of drug targets, treatment, and prognosis.

Proteomics is a comprehensive technology dedicated to the study of all proteins expressed by certain species, individuals, organs, tissues, or cells under certain conditions and within a certain period of time. In 1941, two German scientists, Williams and Wilkin, first proposed the concept of proteome, using this noun method to represent the constituent parts of cells, tissues, or biological proteins [1]. At present, proteomics has been widely used in many fields, and its research content mainly includes two aspects: the study of protein expression patterns and the study of proteomic function patterns [2]. At present, its core technology mainly includes three types: two-dimensional electrophoresis technology (2-DPACE), protein mass spectrometry, and protein identification through database search. The core is mass spectrometry technology, which roughly means that after digesting a pure protein with trypsin, the peptide fragment is obtained according to its deflection and displacement in the electric field to determine its molecular weight and charge, and then the characteristics of all peptide fragments are combined with the database. Knowing the protein for comparison, you can confirm the identity of the protein. In this way, after detecting all proteins in a sample, the detailed information of the proteome of this sample can be obtained [3].The core is a mass spectrometry technology, which roughly means that after digesting a pure protein with trypsin, the peptide fragment is obtained according to its deflection and displacement in the electric field to determine its molecular weight and charge, and then the characteristics of all peptide fragments are combined with the database. Knowing the protein for comparison, you can confirm the identity of the protein. In this way, after detecting all proteins in a sample, the detailed information of the proteome of this sample can be obtained.

RETRACTED

This article discusses myocardial proteomics and its role in sports and related applications. In the process, I consulted a lot of related materials. Among them, Pollastri studied the changes in the hydration state of myocardial protein through the Bioelectrical Impedance Vector Analysis (BIVA) technology and evaluated its impact on the intensity of physical exercise. The results showed that changes in the myocardial proteome can effectively reflect the intensity of physical exercise on the heart and human health [4]. In his research, Shi used high-throughput RNA-seq technology to study the mRNA of myocardial proteins, which confirmed the effectiveness of proteomics at the genetic level and expanded the application of proteomics technology in the field of life sciences [5]. Neunh found in the study that the extension of blood signals can pass through the tight myocardium, which is a unique magnetic resonance (CMR) imaging marker for cardiac magnetic hypertrophy cardiomyopathy or benign congenital malformations. If CMR shows asymptomatic, this may damage to personal health, and the application of proteomic technology can more sensitively detect this signal [6]. Johnson used PAGE and quantified sulfated glycosaminoglycan content (SGAG) to determine the changes in cardiomyocytes in his research and then used ECM targeted quantitative concatemer's (QCONCAT) to analyze by LC-SRM, using 83 representing 48 different proteins. A stable isotope labeled (SIL) peptide quantifies the protein content of myocardium. Quantitative proteomics shows that most of the protein content is composed of various fibril collagen components [7].The protein chip contains the following components: a base, the base has a whole array, a groove on the plate, and the spacer area of the hole on the groove slightly protrudes from the bottom plane of the groove; the reaction body: the reaction body is placed in the recess of the base in the tank, and the reaction body contains a protein reaction membrane; the reaction chamber: the reaction chamber has an array of holes and has a downwardly convex plane, and the convex plane is embedded in the groove of the base to fix the reaction body on the base in the groove.

In the study of myocardial proteomics and its application in sports, this article summarizes and analyzes a large number of previous research experiences and makes some innovations in research content and research methods, mainly as follows: the research mainly used the method of literature investigation to understand the results that have been achieved in the field of proteomics, such as the detection of doping in athletes and early warning of related diseases such as diabetes. With the advent of the genome era, proteomic research has become an important direction for the development of life sciences. Proteomic theory and technology have begun to be applied to research related topics in the field of sports science, and the mechanism of human response and adaptation to exercise plays a role. At the same time, the problems existing in the field of proteomics, such as the effectiveness of proteomics techniques such as quality preservation and the prospects of proteomics, as well as certain explorations and experiments are also discussed. In addition, this rigorous method of controlled experiment is used in the experiment process to ensure the credibility of the research results from the technical level. Finally, this study uses SD rats as a model to explore the application of myocardial proteomics in the field of sports for the first time, providing new ideas for the exploration of proteomics applications.

RETRACTED

## 2. Theoretical Basis of Myocardial Proteomics and Its Role in Sports

### 2.1. Introduction to the Study of Cardiac Proteomics

Myocardial protein is the main part of the heart structure and the direct executor of the pumping function. At the same time, myocardial protein is also an important basis for exercise capacity. Under exercise stress, the expression and conformation of proteins in myocardial tissue change with time and space [8]. Some scientists have used 2-de and maldi-t0f-ms techniques to study the left ventricular by statin in quiet and exercise-trained rats and found significant differential expression of 20 kDa Hsp20 and 3a-hydroxysteroid dehydrogenase [9]. After testing and using the same technique, it was found that, compared with the quiet control group, the increased exercise load after 6 weeks of endurance exercise led to changes in the expression of 26 protein points in the hypertrophic myocardium. In addition, Hsp20 in the myocardium increased significantly after endurance exercise, and the phosphorylation of Hsp20 serine 16 (HSP20-PS16) increased. These studies have shown that endurance training during exercise helps to improve the expression and phosphorylation of Hsp20 in cardiomyocytes. At present, the mechanism of the protective effect of the heat shock protein expression on cardiomyocytes during exercise is still unclear, and further experimental studies are needed.

In different exercise modes, the expression of myocardial proteome is not completely the same. Some scholars have used proteomic technology to study the left atrium, right atrium, and right ventricle of rats after treadmill exercise with different intensities and patterns and identified the cardiac. A-myosin heavy chain, tropomyosin-1, and mannan proteins, some of which are target proteins, have not been involved in research in the field of sports science. These differentially expressed proteins provide a certain experimental basis for further research on new target proteins with sport fatigue characteristics [10]. The highly selective enrichment of a specific target protein in a complex sample is of great significance in the fields of life sciences, clinical testing, food safety, etc. Antibody technology, as the most classic and most mature target protein enrichment technology, is compatible with myocardial protein, and the relationship between them is complementary. In addition, some researchers used 2-DE and MALDI-T0F-MS to increase the load of the left ventricular and right ventricular muscle proteome map of rats after treadmill exercise and found that the differential expression after exercise was more than 10 times that of protein. Some of these identified proteins can be divided into mitochondrial oxidative metabolism, blood pressure regulation, signal transduction, and myocardial oxidative stress based on their characteristics.

RETRACTED

In recent years, some scientists have studied the left ventricular muscle of rats with myocardial infarction after 8 weeks of endurance treadmill exercise through proteomics and western blotting and found that compared with the control group, the left ventricular function of the experimental group of rats has a certain improvement. At the same time, it was found that the expression levels of three specific proteins have changed; that is, the voltage-dependent anion channel 2 (VDAC2) level has decreased. These changes may explain the improvement of myocardial function in rats and provide evidence for studying the molecular mechanism of exercise to improve cardiac function. The study of target proteins in the myocardium under exercise stress is of great significance. Therefore, it can provide an experimental basis for the action and mechanism of myocardial exercise at the proteomics level. This discovery laid the foundation for the preliminary work and provided a reliable basis for further myocardial function research, provided new ideas for cardiac exercise in sports medicine, clinical medicine, etc., and has great medical significance.

### 2.2. Application of Proteomic Technology in Sports

A large number of experiments have proved that proteomic technology, as a key technology in the field of life sciences, has broad development prospects in solving sports science-related problems, there have been researches that have made some progress in these aspects, and the progress is mainly concentrated in the following directions. First, the scientists used MALDI-TOF-MS mass spectrometry to study the proteome of the cardiac muscle of exercise-fatigue rats and identified 10 different proteins, of which 2 proteins were upregulated and 8 proteins were downregulated [11]. Among these proteins, the decrease of four proteins is directly or indirectly related to the body's exercise fatigue, and the increase of only two proteins is clearly related to the degree of body fatigue. These findings will help people understand the molecular mechanisms of human fatigue after exercise. With the lack of protein in the body, muscle mass will gradually decrease, and fatigue is often felt; even if there is enough sleep, it cannot be relieved, and it is accompanied by unresponsiveness. Protein is the main component of hemoglobin. Studying the changes in the expression of skeletal muscle proteome in rats with exercise-induced fatigue, it will be found that the expression of the protein myosin light chain solution and myosin light chain 1 and the protein expression is composed of 9 including glyceraldehyde 3 phosphate dehydrogenase and creatine kinase MB chain, ATP-AMP converting enzyme, myosin heavy chain, and actin protein molecules. These findings will provide an important theoretical basis for studying the molecular mechanism of exercise-induced fatigue. The basic technical roadmap of proteomic research is shown in Figure 1.

RETRACTED

As can be seen from Figure 1, proteomic technologies include protein separation, protein purification, protein identification, and other protein technologies. Many of these technologies have been applied to human scientific research in sports and related fields, including gel electrophoresis, immunoassays and western blotting, enzyme-linked immunoassay protein method and PCR technology, etc. PCR technology generally refers to polymerase chain reaction. Polymerase chain reaction (PCR) is a molecular biology technology used to amplify and amplify specific DNA fragments. It can be regarded as a special DNA replication in vitro. The biggest feature of PCR is that it can greatly increase trace amounts of DNA. These methods have injected new vitality and ideas into the development of sports science. Some scholars have used gel electrophoresis technology to measure the expression of heat shock protein in rat cardiomyocytes after exercise at different periods and intensities and found that exercise can cause the expression of heat shock protein HSP72mRNA in cardiomyocytes to show a sharp increase trend. mRNA generally refers to messenger RNA. Messenger RNA, the Chinese translation of “messenger ribonucleic acid,” is a type of single-stranded ribonucleic acid that is transcribed from a strand of DNA as a template and carries genetic information that can guide protein synthesis [12]. In addition, scientists have studied the effect of exercise on the blood circulation levels of the inflammation-related protein interleukin soluble surface cytoskeleton in patients with overweight/obesity, impaired glucose tolerance, and found that patients with overweight/obesity impaired glucose tolerance expressed abnormal inflammatory factors. Exercise intervention can significantly change this, indicating that proteomics can accurately reflect the protein changes of patients before and after exercise, and provide a favorable, reliable, and convenient basis for disease tracking and treatment.

RETRACTED

In addition, some studies have shown that sport can effectively promote GLU-4 to promote the absorption and utilization of glucose in insulin-deficient rats [13]. Serum cardiac troponin 1 (cTn1) is a serum enzyme with good sensitivity and high specificity. The successful detection of serum troponin 1 helps people distinguish human heart muscle damage from skeletal muscle damage. According to reports, many studies on the changes of serum cardiac troponin 1 before and after swimming in mice indicate that serum cardiac troponin 1 is a good sign of myocardial injury. Someone used enzyme-linked immunosorbent assay to detect the changes in serum cardiac troponin 1 in rats before and after exercise and found that serum troponin 1 in rats did not increase after normal load exercise, indicating that normal intensity load exercise has no effect on cardiomyocyte. This study was found to have great value for the application of proteomics in human sports health research. In addition, a study has long tracked the correlation between the human body's production of plasma stress protein in baseball players and the risk of coronary heart disease and found that among people with high levels of stress protein, 10% to 20% of people may suffer later, such as the development of coronary artery disease and heart disease. Other scholars have used PCR technology to study the polymorphism of the ACE gene, the relationship between angiotensin peptides, endothelin synthase and angiotensin receptors, and the relationship between hypertension and the cardiovascular system of the “athlete heart” and the relationship between functions. In addition, proteomic technology has been widely used to study the relationship between serum CK and lactate dehydrogenase and exercise time and intensity.

RETRACTED

### 2.3. Prospects for the Application of Proteomic Technology in Sports

Due to the establishment of proteomics and the development and maturity of protein chip technology, it can be expected that the research of sports science will be greatly promoted. In the future, scientists may conduct substantive research on exercise and human adaptation at the molecular level. Therefore, the concept of “sports proteomics” may emerge and study the mechanism of human exercise adaptation from the following aspects. First, proteomics can be used to screen nutritional supplements needed by athletes. As we all know, reasonable nutrition supply is not only an important aspect to ensure athletes' health and athletic ability but also a key factor affecting athletes' physical fitness and physical fitness. At present, as a powerful means outside of training, reasonable and scientific nutritional supplements are increasingly favored and concerned by coaches, athletes, and sports researchers at home and abroad. It is conceivable that it is completely possible to use proteomic technology to screen and identify phytochemicals with biological activity and prevent chronic sports diseases and aging. In addition, people can also screen specific markers and nutritional supplements according to the different sensitivity of each athlete to nutritional deficiencies, to determine or predict the high risk of certain sports diseases in certain populations in the future. Therefore, the application of nutritional proteomics and proteomic technology will help develop some healthy (functional) foods that are highly targeted, effective, and high-tech for athletes.

The protein chip technology of proteomics will become a favorable weapon in the fight against doping. In the future, doping in sports can be detected by protein chips. There are two main types of methods: the first is to use antibody chips for detection. This chip can theoretically achieve rapid high-throughput doping detection. However, in many cases, the relative molecular mass of the doped substance is very small, the success rate of preparing specific antibodies is very low, and the cost of this technology is relatively low; so, the research prospects are average. The second method is to use microfluidic separation chip technology, that is, to achieve sample separation, chromatographic identification, mass spectrometry detection, sample electrophoresis, and other chemical analysis methods through the microfluidic device and integrate them in the laboratory on the chip. In recent years, the phenomenon of youth drug use has received widespread attention. The development and research of rapid doping detection technology platforms have not only contributed to the health of competitive sports and athletes but also greatly benefited youth's public health and drug abuse. It will also provide strong technical support for drug management and drug testing. In addition, protein chips can not only detect related stimuli in drugs but even “gene stimuli” cannot be immune. The introduction of foreign genes will inevitably change the expression profile of proteins. Therefore, the establishment of the athlete muscle proteome database will provide a reference and basis for the screening of gene-doped protein chips.

RETRACTED

Through the study of myocardial proteomics, it is expected to reveal the mystery of myocardial protein in sports training, widely play the role of myocardial protein research under different exercise states, establish various sports and sports proteomic databases, and reveal different sports treatments of human physiological functions and movement mechanisms. Through the symbolic proteins of different sports events and exercise loads, it provides direct clues for the evaluation of exercise load and body function in exercise training and provides a theoretical basis for establishing scientific exercise prescriptions for individual exercise fitness and timely monitoring of fitness status. It is to fuse the target protein or polypeptide with the DNA sequence of another protein or polypeptide fragment and express it in bacteria. Fusion expression vectors include secretory expression vector, expression vector with purification tags, surface expression vector, and expression vector with partners. Therefore, they can state and adjust the fitness exercise plan. According to the current research focus of exercise science, myocardial proteomic research is expected to be widely used and developed in many fields such as exercise load and physical function evaluation. Due to the different types and quantities of proteins in different body functions, the specific protein markers under different exercise loads and different physical function states can be found through the establishment of proteomics atlas, and then the exercise load and body function state can be scientifically evaluated. Secondly, proteomics can be used in the selection of athletes: compared with normal physiological processes, athletes of different disciplines show significant upregulation of certain myocardial proteins, while some lack or significantly downregulate. With the advent of the era of big data, the development of high-throughput technology and more sensitive and accurate laboratory instruments have resulted in the continuous expansion of massive proteomic data. The ensuing proteomic database is linked to the Internet, providing molecular biologists with unprecedented opportunities and unlimited use of these information resources. And most of the online proteomic informatic database information resources can be searched or downloaded for free, which greatly promotes the research of proteomics in our country.

RETRACTED

### 2.4. Sports Data Fusion Algorithm

With the increasing complexity of the target environment, the requirements for environmental information and sensor observation accuracy are getting higher and higher, which promotes the emergence and use of various types of multiplatform sensors in sports events. Sensor information fusion technology is a new interdisciplinary subject, and this technology has a wide range of applications in many fields. As an application of information fusion technology in the field of target tracking, multisensor target tracking organically synthesizes multiple sensor information to improve the accuracy of target motion state estimation [14, 15]. The so-called multisensor information fusion is the use of computer technology to automatically analyze and synthesize information and data from multiple sensors or multiple sources under certain criteria to complete the required decision-making and estimation information processing process. Compared with any single sensor target tracking, its tracking accuracy and performance are better and excellent. In proteomic research, if high-throughput methods are used, a large amount of protein data will be obtained, which requires the use of bioinformatic methods for processing. Data fusion technology is an information processing technology that uses computers to automatically analyze and synthesize a number of observational raw data obtained in time series under certain rules to complete the required decision-making and evaluation tasks and process the raw data into advanced data. Data fusion technology can effectively reduce redundant information and reduce the impact of deployment environment through the fusion of node data and obtain a complete and accurate description of the monitoring target [16]. We can obtain the human motion image data and the original data of the motion attitude instrument through the camera and the attitude instrument. These data cannot be understood by people without processing and processing, and there are also noises in these data. We need to process, identify, and analyze these data and finally obtain the data form of the content required by the user. Data fusion is the process of data analysis, optimization, and synthesis of data acquired by devices such as multiroute sensors and cameras [17]. Through data fusion, basic data can be processed into higher-level data that is convenient for further decision-making and processing. Data fusion technology is currently in the preliminary stage of development. Data fusion-related theories and practical application technologies urgently need further indepth research. The data fusion model is shown in Figure 2.

RETRACTED

As can be seen from Figure 2, multidimensional scaling is a very classic method of dimensionality reduction by processing the dissimilarity matrix between data points in a given high-dimensional data space to achieve the purpose of dimensionality reduction. However, because it is difficult to find the dissimilar matrix of data points in the high-dimensional data space, the realization of this method is more difficult. Researching proteomic data is currently an important work of bioinformatics, and it is also the basic cornerstone of mass spectrometry data retrieval. Aiming at the problem of unstable tracking after target occlusion in complex backgrounds, an algorithm for target tracking by fusing heterogeneous information under the framework of particle filtering is proposed. This method establishes a sound source feature model and a color feature model. The main research on the proteome in bioinformatics is to obtain the hidden biological meaning behind the proteome data through the steps of collection, processing, preservation, and searching. Data fusion is the process of inputting raw data records into sensors and then processing the output data or the next process. The composition of this fusion machine is

(1) $$\begin{array}{c} G=\left\|I_{o},A,\alpha ,I_{b}\right\|/r\left(I_{c}\right), \end{array}$$

(2) $$\begin{array}{c} I_{o}=\left[I_{0},I_{1}\right]\left[f0\right]\left(q^{0}⟶q^{1}\right),\left(q^{2}⟶q^{3}\right). \end{array}$$

*G* is the data fusion machine, *I*_*o*_ is the original data, *I*_*b*_ is the next process, *I*_*c*_ is the output data, *A* is the fusion of multiple algorithms, and the relationship between the algorithms is represented by *α*. Equation (2) is the basic mathematical representation. Assuming that a certain action of sport is regarded as a single input node, the corresponding information entropy function is

(3) $$\begin{array}{c} S\left(i\right)=S\left(f_{1},f_{2},\cdots f_{n}\right)=-\overset{n}{\underset{i=1}{\sum }}f_{i}\chi_{f}, \end{array}$$

(4) $$\begin{array}{c} \varepsilon_{i}=1-S_{i}/\overset{n}{\underset{i=1}{\sum }}S_{i}. \end{array}$$

*S* (*i*) is the uncertainty of the information, *f* is the objective reflection of the facts, *f*_*n*_ is the information data carried by the node, and *χ* is the entropy weight. And *ε*_*i*_ is the calculation formula defined by the weight of the monitoring result, and the probability vector to obtain the whole data fusion result is

(5) $$\begin{array}{c} X=\left(x\left(s_{1}\right),x\left(s_{2}\right),x\left(s_{3}\right)\right), \end{array}$$

(6) $$\begin{array}{c} x\left(s_{1}\right)=\overset{n}{\underset{i=1}{\sum }}\eta_{i}x_{i}\left(s_{1}\right), \end{array}$$

(7) $$\begin{array}{c} X\left(s_{n}\right)=\overset{n}{\underset{i=1}{\sum }}\eta_{i}x_{i}\left(s_{n}\right). \end{array}$$

*X* is the probability vector of the data fusion results corresponding to different motion actions, *η*_*i*_ is the node that meets the similarity, and *n* is the number of nodes participating in the data fusion. The calculation formula of the probability of the mean vector within the group can be expressed as

(8) $$\begin{array}{c} {\bar{b}}_{i}=\left({\bar{b}}_{i}\left(s_{1}\right),{\bar{b}}_{i}\left(s_{2}\right),{\bar{b}}_{i}\left(s_{3}\right)\right)=\frac{1}{\text{mm}}\overset{\text{mm}}{\underset{i=1}{\sum }}b_{i}, \end{array}$$

(9) $$\begin{array}{c} l_{i}=\sqrt{\frac{1}{2}\left(\left|s_{i}\right|+\left\|\overset{-}{b_{i}}\right\|+\left(s_{i},{\bar{b}}_{i}\right)\right.}. \end{array}$$

The entropy weight fusion algorithm is used to fuse the node data that meets the similarity condition, the group fusion data ${\bar{b}}_{i}$ is obtained, and the group fusion data replaces the monitoring data of the node *s*_1,2,3,⋯*n*_ in the group to participate in the intracluster fusion. *l*_*i*_ is the mean distance of nodes. Analyze network energy consumption during data fusion processing:

(10) $$\begin{array}{c} l\left(a,b\right)=\sqrt{{\left(s_{a}-s_{b}\right)}^{2}+{\left(q_{a}-q_{b}\right)}^{2}}/\varphi \times e, \end{array}$$

(11) $$\begin{array}{c} E_{i}\left(b,q\right)=\phi ⊗\left(b+q\right)\times l^{3}\left(a,b\right). \end{array}$$

The fusion energy consumption coefficient is 1, and the agent length is *φ*; *φ* × *e* is the energy consumption calculation method of node receiving/sending. The data fusion process is the recognition process of sports images, and the recognition framework of the target image is constructed; there are

(12) $$\begin{array}{c} \underset{i\in w}{\sum }n\left(I\right)=1, \end{array}$$

(13) $$\begin{array}{c} T\left(I\right)=1-\delta \left(\overset{-}{I}\right)=\underset{\delta \cap I\neq \lambda }{\sum }n\left(H\right). \end{array}$$

*n* (*I*) is the basic probability function of image pixel allocation. When there is a decision error in the recognition process, it is *n* (*H*). Calculate the conflict between the two, and then there is

(14) $$\begin{array}{c} n\left(I\right)=\left(n_{1}⊗n_{2}\right)\left(I\right)=\frac{\sum_{I_{1}\cap I_{2}-I}n\left(I_{1}\right)n\left(I_{2}\right)}{1-k}. \end{array}$$

When *k* ≠ 1, *n* (*I*) determines a probability function.

RETRACTED

## 3. Study on the Role of Myocardial Proteomics in Sports

### 3.1. Purpose of the Experiment

The purpose of this article is to study the role and application of cardiac proteomics and related technologies in sports. There are many researches on proteomics and related technologies in the field of sports science. The limitation is that most of the research focuses on urine proteomic research and skeletal muscle proteomic research. There are not many known applications of myocardial proteomics and related technologies in sports, and the research of myocardial proteomics is essential in many diseases. In recent years, reports have found that myocardial cell proteomics research can more accurately reflect the health of the heart and the human body. Especially for athletes, myocardial proteomics research can reflect the load of the heart before and after exercise and related nutrition and provide supplementary needs. Therefore, this research is dedicated to the study of cardiac proteomics and related technologies, including the application and development prospects of protein qualitative and quantitative technologies such as western blotting, enzyme-linked immunoassay, and protein isotope labeling. In the field of sports science, and for the cause of human health and the nutritional supplement, the plan provides an experimental reference and scientific basis.

This article will start from the perspective of myocardial proteomic technology and its application in sports. In previous studies, urine proteomic research, skeletal muscle proteomic research, and other research methods and ideas will be guided to explore myocardial proteomics and learn the application and unique advantages in sports. In the process of research, this research will draw on the research experience of predecessors, while not forgetting to innovate. The main methods used are two experimental methods, such as literature survey and controlled experiment. Firstly, through literature surveys, we will understand the achievements in the field of proteomics, such as the detection of doping in athletes and early warning of related diseases such as diabetes. At the same time, we will understand the current problems in the field of proteomics, such as ensuring the effectiveness of proteomics technology, the prospects of proteomics, and certain explorations and experiments on this. In addition, this rigorous method of controlled experiment is used in the experiment process to ensure the credibility of the research results from the technical level. In summary, the main objectives of this study are twofold: first, introduce the current research progress of proteomics and related technologies and understand the current application prospects and application problems of proteomics, and secondly, study the development and related problems of cardiac proteomics and the application and the role of technology in the field of sports science, based on experiments to achieve certain results, and combined with previous research results to introduce the application prospects and unique advantages of myocardial proteomics and related technologies in the field of sports science. The test structure of the myocardial proteomic exercise model is shown in Figure 3.

RETRACTED

### 3.2. Experimental Materials

Experimental animals: 30 normal male SD rats (body weight of 200 ± 20 g), purchased from Beijing Waiting Lihue Experimental Animal Co., Ltd. (license number: SCXK (Beijing) 2012-0001), were raised in separate cages in the academy of sciences, SPF animal room of the hospital.

Main reagents and instruments are as follows: bromophenol blue, ethylenediaminetetraacetic acid, sodium lauryl sulfate, tris, agarose, Coomassie brilliant blue, and standard protein markers. Antibodies: primary antibodies: Anti-GRP75 antibody, Anti-ATP5A anti-body, and Anti-N calphostin antibody were purchased from Abcam, USA. Secondary antibodies: goat anti-mouse and goat anti-rabbit were purchased from Beijing Zhongshan Jinnia Company. The main instruments used in this study are color Doppler ultrasound imager (model: HP5500, American PHILIPS company), vertical electrophoresis tank (model: Protean Micelle, American Bio-Rad company), gel analysis software (model: Imagemaster2D), American AMER sham Bioscience company), and gel imaging analysis system (model: Gel Doc XR+, American Bio-Rad company).

### 3.3. Experimental Method

Establish a rat model: ligate the anterior descending branch of the left coronary artery to establish a rat model after myocardial death. Three days after the operation, 200,000 units of penicillin were injected to fight the infection. Grouping and administration: 5 days after purchase, animals are fed standard synthetic feed, and 12 hours after fasting, they receive adaptive feed. According to the balance of body weight, the animals were randomly divided into the operation group, sham operation group, and model group, 10 in operation group, 10 in sham operation group, and 10 in model group. Model rats in the model group according to the method were described in the method of animal model replication [18]. After grouping, the rats were given drugs by gavage once a day for 8 weeks. The separation of myocardial mitochondria: differential centrifugation was used to extract myocardial mitochondria. At the end of the 8th week after modeling, the rats were anesthetized, and their hearts were quickly removed by open thoracotomy. Wash the heart repeatedly with PBS buffer, weigh 100 mg of myocardium, add 1.5 mL of homogenate, and homogenize in an ice bath, centrifuge at 1300 r/min for 15 min at 4°C, and save the supernatant. Repeat this procedure twice.

RETRACTED

Extraction of myocardial mitochondrial protein: add 1 mL of lysis solution to the abovementioned myocardial mitochondrial sample, vortex, shake, and break. Place the protein sample in an ice bath for more than 4 minutes to dissolve as much as possible. Two-dimensional gel electrophoresis: take 0.8 mg protein sample, dilute to 350 L with swelling buffer, and mix well. Add the above sample mixture to the side of the bubble expansion box of the bubble expansion plate, put the adhesive strip into the bubble expansion plate, and hydrate for 12 hours. After the hydration is completed, take out the test strip and perform focusing electrophoresis in an isopoint focusing device with the temperature set at 20°C. The temperature setting steps of the isopoint concentrator are shown in Table 1.

Image scanning and analysis: the stained gel is transmitted through the UMAX Power Look2100XL scanner to obtain an image. After scanning, we use imagemas-Ter2D Platinum 5.0 software to detect protein spots, subtract the background, perform matching, standardize, and manually proofread the gel map to find protein spots with differential expression [19, 20]. Western blot verification: differential centrifugation was used to extract myocardial mitochondrial protein from rats. After taking 50 g of the protein sample and sealing it on a shaker for 2 hours, incubate the hybrid primary antibody overnight at 4°C. The membrane was washed, and the hybrid secondary antibody was washed on a shaker at room temperature for 2 hours. Soak the film in an ECL fluorescent lamp for 5 minutes, take it out, and expose it. After scanning exposure, we use GELDOC imaging system to analyze the target zone of the film.

## 4. Results and Discussion of the Myocardial Proteomics and Its Role in Sports

### 4.1. Analysis of Myocardial Proteomic Results

Analysis of the results of two-dimensional gel electrophoresis: in each group, select a gel with high resolution and better quality as the reference gel and match the protein spots among the three gels in the group. If the sample is found to have good repeatability and stable preparation, it can be used for the analysis of different protein spots. After identifying the different protein spots by mass spectrometry, 20 of them were found to reverse the trend of differences. After searching the PMF map data through the Swissport database, 4 proteins were successfully identified. These four proteins are mainly related to human energy metabolism, human stress response, and oxidative damage of cells and tissues. The specific conditions of the four proteins identified are shown in Table 2.

RETRACTED

Research has found that the detection and monitoring of sports biochemical indicators can diagnose the athlete's ability to withstand the load of sports training accurately and timely understand the athlete's physical function reasonably arrange and adjust the training plan, avoid excessive fatigue, reduce sports injuries, and improve sports performance to the maximum to extend. Searching for new biochemical indicators that can reflect the functional status of athletes in a noninvasive, fast, and accurate way has always been the focus of sports research. Therefore, these specific proteins related to athletic ability can be used as biomarkers to provide an objective basis for the selection of new indicators for athletes. In this study, the left ventricular ejection fraction, left ventricular short axis shortening rate, and left ventricular diastolic end diameter were compared. The specific data are shown in Figure 4.

It can be seen from the data in Figure 4 that among the three groups of rats, the left ventricular ejection fraction of the sham operation group was the highest, which was 7.7% and 4.6% higher than that of the operation group and the model group, respectively. The short axis of the left ventricle of the operation group was shortened. The short axis of the left ventricle of the operation group was shortened, the highest rate and the longest left ventricular diastolic inner diameter.

Research results show that the most important application of cardiac proteomics is the detection of stimulants in exercise. Proteomics studies the characteristic protein markers caused by different stimuli to detect the use of stimuli. The training model of the data network unit of cardiac proteomics in motion is constructed in conjunction with the human heart, as shown in Figure 5.

Proteomics can also provide a basis for exercise prescription or the development of innovative exercise training methods. Through the study of myocardial proteomics, we explore the characteristics of myocardial protein components for optimal exercise and fitness, then determine the exercise goal, develop innovative exercise training methods, and choose exercise time according to physical function conditions to guide exercise training and exercise fitness. The results of the study of myocardial protein components can also be used to make protein chips with different functions, thereby simplifying the operation of various experiments. Since fatigue markers (enzymes or peptides) are selected in the myocardial protein components and then made into receptors or enzyme chips, the athlete's myocardial protein samples will be labeled after the reaction of the chip, and high-throughput parallel detection of fatigue markers can be performed at the same time, determine the degree of recovery or fatigue, and coordinate the training plan. In this study, the resting cell length, maximum contraction velocity, and peak time of the three groups of rat cardiomyocytes were recorded. The specific data are shown in Figure 6.

RETRACTED

It can be seen from the data in Figure 6 that among the three groups of rats, the myocardial cells in the operation group are the longest, 1.3% and 14.7% higher than those in the operation group and the model group, respectively. The maximum contraction speed of myocardial cells in the model group is the fastest, 13.7% and 16.2% higher than the rats in the operation group and the sham operation group, respectively. The rats in the sham operation group have the longest peak time. This shows that myocardial proteomics can accurately reflect the heart condition of rats.

### 4.2. Discussion on the Advantages of Myocardial Proteomics in Sports

The application of myocardial proteomics in sports has certain advantages. The study of myocardial mitochondrial proteomics is expected to find some target proteins related to the pathogenesis of myocardial ischemia-reperfusion injury (IR). The analysis of the functional pathways of these target proteins is of great significance for further revealing their mechanisms. The 2-DE technology in myocardial mitochondrial proteomic research has high requirements for sample preparation. The sedimentation coefficients of cytoplasmic proteins, endoplasmic reticulum, and microsomes are similar to those of mitochondria; so, it is difficult to separate them completely by differential centrifugation. Sample purity is the key to the success of myocardial mitochondrial proteomics. At present, mitochondria are mainly extracted by differential centrifugation, but it is difficult to separate components with similar sedimentation coefficients. These nonmitochondrial components will seriously affect the effect of isoelectric focusing, which may prevent a small amount of protein from entering the IPG band. Therefore, this study has made corresponding changes in the references. The mitochondrial separation medium was used to replace the pediocin dissolved in sucrose to maintain the osmotic pressure of the mitochondria, and the centrifugal speed was changed from 52,000 r per 90 minutes to 100,000 r per 60 min. Western blotting results showed that the mitochondria obtained by density gradient centrifugation had higher purity. In this experiment, after 2-DE, the gel was stained with silver nitrate and centrifuged by density gradient to make the purified gel image clearer and the background clearer. All selected protein spots were identified as mitochondrial proteins by mass spectrometry, indicating that the sample preparation method used in this experiment is reliable. This study investigated the application of proteomics in the field of sports science. The specific results are shown in Figure 7.

RETRACTED

From the data in Figure 7, it can be seen that the application of myocardial proteomics in the field of sports science shows a diversified trend, mainly including doping detection, accounting for 28%, sports selection, accounting for 27%, nutritional supplementation, accounting for 25%, sports classification, accounting for 12%, and prevention sensitive, accounting for 8%.

Ligating the left anterior descending artery of the rat after myocardial infarction is one of the methods to establish a myocardial animal model. According to the results of this experiment, the heart rate of the rats before the intervention was normal, the breathing was steady, and the activity and mental state were not affected. The increase in heart rate of rats in the model group reflects the symptoms of palpitation, and the shortness of breath reflects the symptoms of shortness of breath and wheezing. Reduced activity, lethargy, withered and yellowed hair, raised resistance and resistance, and other general conditions reflect the expression of symptoms such as fatigue, lack of breath and lazy speech, lips, tongue, and nails with dark purple reaction to blood stasis syndrome. Therefore, the model established in this study can better reflect the characteristics of exercise-related syndromes and can be used as an animal model for exercise effects. In this study, it was observed that after surgical intervention, the model rats' heart rate slowed down, shortness of breath, decreased activity and mental state, food intake, dark purple lips, and tongue, but did not improve the prognosis and insufficient blood stagnation. In scientific statistical analysis, this is the lack of perfection in this experiment. This study investigated the length, diastolic velocity, and diastolic time of three groups of rat cardiomyocytes. The specific data are shown in Figure 8.

It can be seen from Figure 8 that the cardiomyocyte length, diastolic velocity, and diastolic time of the three groups of rats are different. Among them, the cardiomyocytes of the operation group are the longest, and the diastolic time is the longest, which are higher than those of the sham operation group and the model group. 37.1% and 8.5%: the model group has the highest diastolic velocity. The length of the cardiomyocytes of the three groups of rats is between 85 and 90, the diastolic velocity is between 57 and 82, and the diastolic time is between 72 and 95.

RETRACTED

## 5. Conclusions

1. This research first introduces the current research progress of proteomics and related technologies, understands the current application prospects and application problems of proteomics, and secondly, studies the development of myocardial proteomics and the application and role of related technologies in the field of sports science. Based on the experiments, certain results have been obtained, and combined with previous research results, the application prospects and unique advantages of myocardial proteomics and related technologies in the field of sports science are introduced. In view of the importance of the heart in sports science, applying myocardial proteomics to sports science and studying the changes of myocardial proteomics under exercise stimulation at an overall level will undoubtedly greatly promote the development of sports science
2. The results of the study showed that among the three groups of rats, the left ventricular ejection fraction of the sham operation group was the highest, which was 7.7% and 4.6% higher than that of the operation group and the model group, respectively. The operation group had the highest left ventricular short axis shortening rate, while the left ventricle has the longest diastolic inner diameter. In addition, among the three groups of rats, the myocardial resting cells in the operation group were the longest, 1.3% and 14.7% higher than those in the operation group and the model group, respectively. The maximum contraction speed of myocardial cells in the model group was the fastest, which was higher than that in the operation group and the model group. Rats in the sham operation group were 13.7% and 16.2% higher, respectively. The rats in the sham operation group had the longest peak time. It can be seen that myocardial proteomics can accurately reflect the heart condition of rats
3. The research in this paper shows that the length, diastolic velocity, and diastolic time of the three groups of rat myocardial myocytes are different. Among them, the myocardial cells of the operation group are the longest, and the diastolic time is the longest, respectively, compared with the sham operation group, and the model group was 37.1% and 8.5% higher, and the model group had the highest diastolic velocity. In addition, the application of myocardial proteomics in the field of sports science shows a diversified trend, mainly including doping detection, accounting for 28%, sports selection, accounting for 27%, nutritional supplements, accounting for 25%, sports classification, accounting for 12%, and prevention of sensitivity, accounting for 8%.

RETRACTED

## Figures and Tables

**Figure 1:** Basic technology roadmap for proteomic research.

**Figure 2:** Data fusion model.

**Figure 3:** Myocardial proteomics exercise structure.

**Figure 4:** Comparison of left ventricular ejection fraction, short-axis shortening rate, and end-diastolic diameter in the three groups of rats.

**Figure 5:** Sports training data unit structure.

**Figure 6:** Changes of resting cell length, maximum contraction velocity, and peak time of three groups of rat cardiomyocytes.

**Figure 7:** Main applications of cardiac proteomics in the field of sports science.

**Figure 8:** Comparison of the length, diastolic velocity, and diastolic time of three groups of rat cardiomyocytes.

**Table 1:** Temperature program setting of isopoint focusing instrument.

Step	Voltage/V	Voltage time product/Vh
S1	0-500	500
S2	500	2500
S3	500-3500	10000
S4	3500	50000

**Table 2:** 4 successfully identified proteins.

Accession no.	Molecular mass	Sequence coverage	Mascot score
GRP75-MOUSE	73461	21	54
OAT-MOUSE	48324	19	67
GSTP2-MOUSE	25687	43	89
DHE3-MOUSE	62298	21	68

## Data Availability

The data underlying the results presented in the study are available within the manuscript.
